# Obstructive Sleep Apnea Syndrome Treated Using a Positive Pressure Ventilator Based on Artificial Intelligence Processor

**DOI:** 10.1155/2021/5683433

**Published:** 2021-09-23

**Authors:** Zhuxiang Chen, Zhang Zhao, Zhimin Zhang

**Affiliations:** Hubei No. 3 People's Hospital of Jianghan University, Wuhan 430033, Hubei, China

## Abstract

With the acceleration of people's life rhythm, obstructive sleep apnea syndrome appears more and more frequently. This research mainly discusses the treatment of obstructive sleep apnea syndrome with a positive pressure ventilator based on artificial intelligence processor. The information storage function of the smart positive pressure ventilator is included in the local medical terminal, presented after logging in with the user authority. It is mainly composed of data collection, data processing, and medical interface design, which embeds data request, data transmission, data analysis, and detailed tasks such as data compression and storage, and functions such as data display, image drawing, and alarm notification are realized by the medical interface. When the CPAP ventilator transmits respiratory data to the local medical terminal, it sends real-time respiratory information data packets. The data packet is collected and sent in real time in a fixed period and then received and analyzed by the local medical terminal. In the CPAP ventilator telemedicine system, the function of alarm message processing is mainly used to detect the patient's breathing status in real time, extract the alarm-related information, and generate an alarm. This function specifically includes several tasks such as alarm detection, alarm prompt, alarm storage, and remote transmission of alarm messages. The confirmed OSAS patients were pressure-titrated with a smart CPAP ventilator and then treated for 5 hours a day, followed by echocardiography after 5 months of continuous treatment. During the study, the average BMI was (28.9 ± 7.2) kg/m^2^ and the average AHI index was (53.1 ± 37.8) times/h. This study may help improve the quality of life of patients with obstructive sleep apnea syndrome.

## 1. Introduction

Many studies have shown that OSA is a heterogeneous disease, and its clinical characteristics, pathophysiological characteristics, and polysomnography all have different phenotypes. The current clinical guidelines for assessing the severity of OSA and the main indicators of treatment effects are still based on the assessment of AHI and blood oxygen saturation in polysomnography, although there are a large number of studies on OSA-related biomarkers, endothelial function, and arterial stiffness in the literature; although there are a large number of research evaluations on OSA-related biomarkers, endothelial function, and arterial stiffness in the literature, there is no clinical practice guidance.

The use of medical information technology has become an important way to improve the level of medical services and medical quality [1]and are the key factors that influence the adoption of medical information technology and related applications by adopters. CPAP can significantly reduce the prevalence of MS during the treatment of OSAS but has limited impact on BMI; a healthy and reasonable diet can effectively control weight and reduce the prevalence of OSAS, MS, and other related metabolic indicators.

Artificial intelligence (AI) has promoted the development of today's technology. Sharaf El Din et al. believe that due to the existence of various pollutants produced by human, agricultural, and industrial activities, the quality of surface water has deteriorated. Their research attempts to develop an artificial intelligence modeling method to plot the concentration of optical and nonoptical SWQP. Although their research can retrieve different SWQP concentrations from Landsat8 images, the research still lacks logic [2]. Hashemi et al. believe that process-based models have been widely used for storm surge prediction. The authors used the high-resolution wave and surge modeling system on the East Coast of the United States to numerically simulate 1,050 tropical storms. Their research provides an unprecedented data set. Although their research can be used to train artificial intelligence models for surge prediction in those areas, the accuracy is not high [3]. Bose believes that these technologies provide powerful tools for modern smart grid (SG) control. His applications include the automation design of modern wind power generation systems and their operating status monitoring under operating conditions, the failure mode recognition of SG subsystems, and the SG control based on real-time simulators. Although the concept of these application examples he proposed can be extended to develop many other applications, there is still a lack of specific data [4]. Raedt et al. studied uncertainty in probability theory and graphical models and studied relationships logically. They focused on two detailed representations: Markov logic network (an expansion of the relationship between undirected graphical models and weighted first-order predicate calculus formulas) and Problog (probability expansion of logic programs), which can also be regarded as Turing complete expansion of the relational Bayesian network. Their research discusses Markov logic networks but still lacks theory [5].

The information storage function of the smart positive pressure ventilator is included in the local medical terminal, presented after logging in with the user authority. It is mainly composed of data collection, data processing, and medical interface design, which embeds data request, data transmission, data analysis, and detailed tasks such as data compression and storage, and functions such as data display, image drawing, and alarm notification are realized by the medical interface [6]. The data packet from the CPAP ventilator is collected and sent in real time in a fixed period and then received and analyzed by the local medical terminal. In the CPAP ventilator telemedicine system, the function of alarm message processing is mainly to detect the patient's breathing status in real time, extract the alarm-related information, and generate an alarm. This function specifically includes several tasks such as alarm detection, alarm prompt, alarm storage, and remote transmission of alarm messages. The confirmed OSAS patients were pressure-titrated with a smart CPAP ventilator and then treated for 5 hours a day, followed by echocardiography after 5 months of continuous treatment.

## 2. Treatment of Obstructive Sleep Apnea Syndrome

### 2.1. Artificial Intelligence

The application of artificial intelligence in the medical field has produced smart medical systems in the early stage, which is the main research and development direction of medical research in the future, and it is also one of the parts that this article focuses on. The impact of technological changes may reform it in two ways. One is that most automated operations will replace workers, which will reduce the number of jobs in the market, loss of job opportunities, and changes in places in the society that require people to perform low-skilled jobs [7]. The inefficiency and cost reduction brought about by these phenomena will eventually create wealth. There is another phenomenon that makes it more difficult to predict. The results of scientific and technological progress will change the rules of the game in the market, because it indirectly makes the merchants on the market reorganize and rebuild their operating methods and operating models. Such market process improvements and organizational changes will cause many jobs, repetitive tasks, and low-skilled personnel to be eliminated. For the field of smart medical care, it is also facing the same problem, but it is gratifying that medical robots or other technological technologies will gradually replace and eliminate low-level, low-skilled, and even overcharged doctors in the market and standardize the smart medical market [8, 9]. According to the results of the questionnaire evaluation, a judgment matrix of *n* evaluation indicators can be obtained, among which *C*1, *C*2, *C*3,…, *Cn* are the evaluation indicator of the medical APP user experience [10].

(1) $$\begin{array}{c} R=\begin{array}{c} C1\\ C2\\ \vdots \\ Cn \end{array}\left[\begin{array}{cccc} a_{11} & a_{12} & \cdots & a_{1n}\\ a_{21} & a_{22} & \cdots & a_{2n}\\ \vdots & \vdots & \vdots & \vdots \\ a_{n1} & a_{n2} & \cdots & a_{nn} \end{array}\right]. \end{array}$$

The negative results of OSA in these studies are not only related to OSA itself but also may be related to the current evaluation indicators for OSA. The importance of the project *C*_*i*_ relative to *C*_*j*_ can be expressed as [11, 12]

(2) $$\begin{array}{c} A_{ij}=\frac{w_{i}+1}{w_{j}}. \end{array}$$

The existing intelligent medical auxiliary diagnosis system ignores the relationship between doctors and patients and does not take into account the influence of factors such as system information quality and risk, which is not conducive to the further development of intelligent medical care. However, the traditional intelligent medical‐assisted diagnosis and decision‐making methods are weak in processing multimodal data. There is a lack of research on methods of auxiliary diagnosis and decision‐making based on multimodal data, and the various medical data of patients are not fully utilized for diagnosis. In addition, the interpretability of the model is not strong, which makes the output information unfavorable for doctors to understand. To ensure the realization of this medical function, hospital management is indispensable and its determinant *A* can be expressed as [13]

(3) $$\begin{array}{c} A=\left[\begin{array}{ccc} \frac{w_{1}}{w} & \cdots & \frac{w_{1}}{w_{n}}\\ \vdots & \vdots & \vdots \\ \frac{w_{n}}{w_{1}} & \cdots & \frac{w_{1}}{w_{n}} \end{array}\right]*\left[\begin{array}{c} w_{1}\\ \cdots \\ w_{n} \end{array}\right]. \end{array}$$

Although artificial intelligence includes the word “intelligence,” it is mainly an artificial agent that simulates a series of complex activities related to human intelligence such as perception, learning, reasoning, and communication, through computers. The difference between artificial intelligence and human natural intelligence is that its production can save a lot of organic activities such as metabolism and reproduction. Its production is like the realization of human intelligence on a machine. Because the development and use of smart machines can simulate and extend the functions of human organs, they have replaced many simple, repetitive, and even complicated tasks that are difficult to do in ordinary times [14]. Hence, the society's demand for workers has undergone a huge change [15]. Therefore, the evaluation standard *W*_*i*_ is

(4) $$\begin{array}{c} W_{i}=\sum_{j=1}^{n}\frac{a_{ij}}{\sum_{i=1}^{n}a_{ij}},\;i,j=1,2,3,\ldots ,N. \end{array}$$

### 2.2. Positive Pressure Ventilator

Noninvasive positive airway pressure ventilation (NIPPV) includes normal (CPAP) and smart CPAP (Auto CPAP) ventilation and bilevel positive airway pressure (BiPAP) ventilation. For OSAHS patients, maintaining the open upper airway can solve the collapse of the upper airway during sleep, thereby improving sleep apnea and hypopnea and significantly improving the sleep quality of patients. This is especially observed in patients with moderate to severe OSHAS. Patients with severe daytime sleepiness and systemic complications should be treated with continuous positive airway pressure as the first choice. When using noninvasive positive airway pressure, the pressure level should be set, and setting an appropriate pressure can ensure the efficacy [16, 17].

(5) $$\begin{array}{c} v_{id}^{k+1}=\omega v_{id}^{k}+c_{1}\zeta \left(p_{id}^{k}-x_{id}^{k}\right)+c_{2}\eta \left(p_{gd}^{k}-x_{id}^{k}\right),\\ x_{id}^{k+1}=x_{id}^{k}+v_{id}^{k+1}, \end{array}$$

_where_*v*_*id*_^*k*+1^ represents the operating speed of the positive pressure ventilator. *x*_*id*_^*k*+1^ stands for the risk level [18].

#### 2.2.1. Face Mask

The face mask is the part that has contact with the patient during continuous positive pressure ventilation. The choice of the mask should be appropriate, and the patient's comfort affects the patient's treatment effect and compliance with the application of noninvasive positive airway pressure. At present, the types of facial masks include oral-nasal masks, nasal masks, nasal pillows, mouth-mounted, full-face masks, helmets, etc. At present, the most widely used are oral-nasal masks and nasal masks. There are no standardized guidelines for the selection of masks, and the patient's comfort is the main basis for mask selection; besides, the patient's facial shape and presence of facial deformities are also the basis for mask selection.

#### 2.2.2. Mask Humidifier

The mask humidifier is an integral part of the ventilator. At present, all types of ventilators basically have the application of heating and humidifying, which enhances the comfort of patients using the ventilator [19]. The positive pressure ventilator is shown in Figure 1.

### 2.3. Obstructive Sleep Apnea Syndrome

Obstructive sleep apnea hypoxia syndrome (OSAHS) refers to the repeated collapse of the upper airway during sleep, which causes apnea and hypoventilation during sleep, accompanied by snoring, sleep structure disorders, and frequent occurrences of symptoms such as decreased blood oxygen saturation and daytime sleepiness. OSAHS is a common disease that can occur at any age, and genetic factors can increase its incidence by 2–4 times. Due to snoring at night, the patient frequently wakes up, lacks physical strength and energy, and develops sleepiness during the day. OSAHS is also a potential disease that causes damage to the heart and cerebrovascular system [20].

(6) $$\begin{array}{c} f\left(x\right)=\left(\frac{2}{1+e^{-2x}}\right)-1. \end{array}$$

This repeated airway obstruction often exposes patients with OSAHS to intermittent hypoxemia/hypercapnia and sleep fragmentation. There is considerable evidence that, compared with non-OSAHS patients, OSAHS patients have significantly higher morbidity and mortality due to various complications, especially cardiovascular complications [21]. If *T*_*p*_=*p* is estimated on average, it is called unbiased estimation. For unbiased estimation, there is [22, 23]

(7) $$\begin{array}{c} A=\int p\left(z_{1}|p\right)\cdots p\left(z_{m}|p\right)\Delta T\text{d}z_{1}\cdots \text{d}z_{m}. \end{array}$$

Calculating the partial derivative of *p* with formula (7), we get the following [24]:

(8) $$\begin{array}{c} A_{1}=\sum_{i=1}^{m}\int p\left(z_{1}|P\right)\cdots P\left(Z_{m}|p\right)\frac{1}{p\left(Z_{i}|p\right)}\frac{\partial p\left(Z_{i}|p\right)}{\partial P}\Delta T\text{d}z_{1}. \end{array}$$

Biological activity refers to sympathetic nerve activation, metabolic effects, and systemic inflammation. The HbA1C, night blood pressure type, and hs‐CRP were evaluated, and it was concluded that the influencing factors on patients mainly included quality of life, daytime sleepiness, depressive symptoms, attention, and alertness of sexual desire; pathophysiological characteristics include muscle dysfunction, arousal threshold, loop gain, and anatomical factors. The authors used a clinical fingerprint tool to visualize the severity of the disease, biological activity, and the impact on the patient and found that this method can also present different treatment responses, thereby guiding doctors to individualize the treatment of these patients. Because *p* is dependent on *T*_*p*_ instead of *T*, formula (8) can be converted to [25, 26]

(9) $$\begin{array}{c} A_{2}=\int P\left(Z_{1}|P\right)\cdots P\left(z_{1}|P\right)\frac{1}{p\left(z_{i}|p\right)}\left(\sum_{i=1}^{m}\frac{\partial \;\ln\;p\left(z_{i}|p\right)}{\partial p}\right)\text{d}z_{1},\\ E=\frac{\sum_{k=1}^{n}{\left(y_{k}-o_{k}\right)}^{2}}{n}, \end{array}$$

where *E* stands for total effectiveness. According to the main data used by the system, the current smart medical auxiliary diagnosis system on the market is mainly divided into two, one based on medical imaging and the other based on medical text. Among them, the smart medical auxiliary diagnosis system based on medical imaging has become the research hotspot of many enterprises, and it is widely used in the current practical application. In recent years, the academic circles have gradually deepened their understanding on sleep-disordered breathing. If hypoventilation is set as the connection weight between the clarity and the rule layer, *δ*_*i*_^3^, then [27]

(10) $$\begin{array}{c} \delta_{i}{}^{3}=\frac{\partial E}{\partial O^{3}{}_{i}}=\sum_{i=1}^{C}\frac{\partial E}{\partial O_{i}^{4}}\times \frac{\partial O_{i}^{4}}{\partial O_{i}^{3}}\\ =\sum_{i=1}^{C}\frac{\partial E}{\partial O_{i}^{4}}\times W_{ij}\frac{\sum_{k=1}^{\delta }O_{k}^{3}-O_{j}^{3}}{\sum_{k=1}^{\delta }O_{k}^{3}}. \end{array}$$

The human body is a complex biological system, in which OSAS is often associated with metabolic abnormalities [28, 29]. Intermittent hypoxemia and susceptibility to wakefulness may be the key factors that trigger a series of downstream cardiovascular diseases, including sympathetic nervous system activation, inflammation, and oxidative stress. Obesity and visceral obesity are the main risk factors for obstructive sleep apnea. The abnormal indicators such as inflammation, hormones, and binding proteins caused by it may play an important role in the complications of cardiovascular events [30]. Here, *S* is the number of fuzzy rules generated by *δ*_*i*_^3^ [23].

(11) $$\begin{array}{c} H_{p}\left(z\left(t\right)\right)=\frac{\prod_{m=1}^{l}M_{pm}\left(z\left(t\right)\right)}{\sum_{p=1}^{r}{∐}_{m=1}^{l}M_{pm}\left(z\left(t\right)\right)}. \end{array}$$

## 3. Obstructive Sleep Apnea Syndrome Experiment

### 3.1. Smart Positive Pressure Ventilator

The information storage function of this ventilator is included in the local medical terminal, presented after logging in with the user authority. It is mainly composed of data collection, data processing, and medical interface design. It embeds data request, data transmission, data analysis, data compression and storage, and detailed tasks, and the medical interface realizes functions such as data display, image drawing, and alarm prompts.

#### 3.1.1. Data Collection

*(1) Data Communication Mechanism*. In the CPAP ventilator telemedicine system, the RS485 serial interface is used between the CPAP ventilator and the local medical terminal to communicate with the MODBUS protocol. Therefore, serial communication parameter setting, serial port opening, and data receiving and verifying processes must be carried out in sequence. The ultimate goal of realizing the RS485 communication interface is to allow the CPAP ventilator to communicate with the local medical terminal through the serial port. In the serial communication programming, this article adopts the API function that Windows encapsulates to realize.

When the local medical terminal communicates with the CPAP ventilator, the received data is a sequence formed in bytes, so the common look-up table method is used to calculate the CRC-16 check code and the byte sequence is CRC checked.

*(2) Data Communication Protocol*. When the CPAP ventilator transmits respiratory data to the local medical terminal, it sends real-time respiratory information in the form of data packets. The data packet is collected and sent in real time in a fixed period and then received and analyzed by the local medical terminal. At this time, the ventilator model and version number information is filed in the address field, so that it can be mapped to the corresponding ventilator data table in the database during communication.

#### 3.1.2. Data Processing

*(1) Design of Real-Time Database*. Taking into account the design requirements and goals of the system, we finally decided to use Fast DB, an open-source memory real-time database. Fast DB has obvious time advantages in database access and operation. When a new user of CPAP ventilator is added, the program automatically creates a database DB for it and executes record insertion/deletion operations. When the communication starts, the database is opened. Before that, it is necessary to determine whether the database is occupied. If the database is occupied, wait for it to be released before opening. After that, its interface function is used to perform operations such as reading and writing data values. After the communication is over, the database is closed. If you want to delete a user, set the question to ask the database whether to keep existing data.

*(2) Historical Data Storage*. When storing historical data, a lossless compression mechanism based on incremental compression is first used and then the compressed data is inserted into the dat file (in-disk) in the form of a serialized binary file. On the contrary, when reading historical data, first deserialize the dat file and then decompress the obtained data to get the original data.

#### 3.1.3. Design and Realization of Alarm Message Processing

In the CPAP ventilator telemedicine system, the alarm message processing function is mainly to detect the patient's breathing status in real time, extract the alarm-related information, and generate an alarm. This function specifically includes several tasks such as alarm detection, alarm prompt, alarm storage, and remote transmission of alarm messages.

#### 3.1.4. Overall Design of the Interface

In the design of the medical interface of the CPAP ventilator telemedicine system, the basic elements such as the menu bar, the toolbar, the status bar, and the client area are included. The client area is the main function realization area, which is divided into the communication setting area and drawing operations. There are five parts: client area, communication area, image drawing area, value display area, and remote interaction area. The operating principle of the smart positive pressure ventilator is shown in Figure 2.

### 3.2. Smart Breathing Monitoring

Two-way communication of doctor-patient information is done within the cloud platform. After doctors and patients log in to the cloud platform through their respective accounts, they can send and receive each other's emails to achieve online communication within the cloud platform, similar to internal forum emails; the cloud platform sends directly the information to the patient's ventilator screen, and the doctor obtains the data on the cloud platform. After sorting and analyzing, it is found that the patient's ventilator use matters need to be prompted or corrected. The reminder information can be directly pushed to the patient's ventilator screen on the cloud platform. OSAHS patient classification management involves patient groups under the doctors to be classified according to the needs of each doctor for patient management or academic research by the health index value; if there are patients in the classified group that exceed or fall below the preset value, the cloud platform will automatically alert and classify the patient group later and the workload of doctors will be greatly reduced. The cloud platform will automatically push reminders to patients who exceed or fall below the value based on the preset value of group data.

#### 3.2.1. Data Transmission and Preservation Process

The original data is first stored in the ventilator, and the first is to guarantee that it is not lost; it is transmitted to the wireless transmission box through the data line and then automatically uploaded to the cloud by the China Mobile network to achieve secondary storage and calculation. This process involves fully automatic data transmission on the hardware side.

#### 3.2.2. Use Process of Sleep Cloud Platform

Open any computer connected to the Internet, and enter the URL in the browser to log in to the platform; there is no need to download third-party software and perform complicated registration verification. After the account is created by the superior administrator, you can log in to any PC from any place (global) to access the network to browse the required information i.e., 5 kinds of comprehensive reports (summary report, daily report, weekly report, monthly report, compliance report). The summary report contains user information, equipment information, and monthly calendar information overview; daily reports include user information, all-day event information and charts, all-day trend charts (leak, pressure, blood oxygen, pulse rate, etc.); weekly reports, monthly reports, and compliance reports include time-period event overview information, charts, and time cycle compliance diagram (use time, high/low/average pressure, and high/low/average blood oxygen). The cloud platform presents big data in the true sense.

### 3.3. Research Objects

We have selected patients who came to our hospital's respiratory medicine testing room, Ward's sleep testing room, and sleep treatment center PSG from November 2018 to October 2019 to diagnose OSAHS and those who have been treated with a ventilator. All patients received the consent of their family members and signed an informed consent form, and the experimental process was approved by the ethics committee:

1. Patients whose use of CPAP is contraindicated were excluded.
2. Patients with one of the following or a combination of multiple conditions were not allowed to participate in the test: severe infection, insomnia, severe coronary heart disease, and emphysema.
3. Patients with emotional disorders that may affect the test were excluded.
4. Because patients with anxiety and other anxiety emotions such as fear can significantly affect the compliance of CPAP treatment, for OSAHS patients who wanted to participate in the test, the Venham Clinical Anxiety and Cooperative Behavior Rating Scale was measured, and we excluded patients with level 4 (fear) and above from the test.

### 3.4. CPAP Treatment

OSAS patients diagnosed by PSG were given a smart CPAP ventilator to perform pressure titration, the optimal pressure was analyzed, and then treatment was given for 5 hours a day. At the same time, experts would be organized for visits from time to time and echocardiography would be performed after 5 months of continuous treatment.

### 3.5. Statistical Processing

Rev Man 5.0 software was used for statistical processing of data. The correction coefficient *Q* test based on the chi-square test was used to measure whether there is a significant difference in the research process, and the value of the test level *α* is set to 0.10. There is a high degree of heterogeneity between the groups when *P* < 0.10 or *P* > 0.5. If there is clear heterogeneity, descriptive statistical analysis is required. The measurement data was tested by *Z* test and 95% CI, and *P* < 0.05 indicated that the difference was statistically significant.

## 4. Results and Discussion

Among the patients, 3 cases were excluded from the original PSG sleep monitoring report due to nonreporting, 3 cases were excluded due to voluntary withdrawal from the patient, 4 cases were excluded due to the inability to conduct a follow-up visit, and 3 cases were excluded due to incorrect card reading data. A total of 69 cases were included in the final investigation and analysis. There were 53 males and 16 females. The average age was 50 ± 26 years, the average BMI was (28.9 ± 7.2) kg/m^2^, the average AHI index was (53.1 ± 37.8) times/h, and the average machine time was (555.5 ± 463.5) days. The treatment status of each group is shown in Table 1.

Logistic regression analysis of treatment compliance with noninvasive positive airway pressure: taking noninvasive positive airway pressure treatment compliance as the dependent variable, the patient's gender, age, BMI, inconvenience to wear, living conditions, chronic airway disease, systemic comorbidities, ventilator mode, face mask, interval between diagnosis and wearing ventilator, patient health education, patient family health education, follow-up visits, upper airway surgery history, bad habits, adverse reactions, night insomnia symptoms, initial AHI index, the initial LSpO_2_, the AHI index after treatment, and the total number of days of ventilator use were taken as independent variables. The Wald stepwise regression method was used to introduce a logistic regression model. The logistic analysis result is shown in Figure 3.

Among the 87 study subjects, 35 were smokers (40.2%), 41 were obese (47.6%), 24 had hypertension (27.6%), and 33 smokers (37.9%) were treated with CPAP for six months. 37 cases of obesity (42.5%) and 20 cases of hypertension (23.0%), AH decreased after 6 months of CPAP treatment, and the difference was statistically significant (*P* < 0.05); the minimum SaO_2_ increased, and the difference was statistically significant (*P* > 0.05). There was no significant difference in neck circumference, waist circumference, hip circumference, FG, TC, TG, HDL, LDL, dSBP, dDBP, nSBP, nDBP, average SaO2, ODI, heart rate, etc. The changes of each index before and after treatment are shown in Table 2.

The neck circumference (NC) of 73 randomly selected subjects was 30–48 cm, with an average of (40.715 ± 4.421) cm, and the body mass index (BMI) is (17.1–39) kg/m^2^, and the average is (28.292 ± 4.353) kg/m^2^, PSG. The detection result was that the AHI was (1.20–95.80) times/h, and the average was (39.798 ± 25.77) times/h. The correlation equation Pearson correlation coefficient was used to test the correlation between two variables. We compared the correlation between NC, BMI, and AHI, respectively. Comparison between BMI and AHI showed that there is a positive correlation between the two (*β* = 0.504, *P* < 0.05). In the same way, the bivariate correlation between NC and AHI was compared and it was concluded that there was a positive correlation between NC and AHI (*β* = 0.692, *P* < 0.05). At the same time, the greater the *β* value, the greater the correlation between NC and AHI. The measurement results of each index of the subject are shown in Figure 4.

Pearson correlation analysis showed that age, neck circumference, AHI, ODI (depletion of oxygen index), and average SpO_2_ (mean oxygen saturation) were significantly correlated with lactic acid, and the correlation coefficients (*r*) were −0.268, 0.214, 0.213, 0.210, 0.461, and −0.299; the *P* values were 0.005, 0.027, 0.026, 0.028, 0.000, and 0.002, respectively. In addition, age, neck circumference, and PH value were positively correlated, among them, correlation coefficient *r* was 0.378, 0.214, *P* value is 0.000, 0.049 respectively, and ODI was negatively correlated with PH value (*r* = −0.215, *P*=0.025). The Pearson correlation analysis results are shown in Figure 5.

The proportion of men in the moderate-to-severe OSAHS group was higher (*P*=0.001), and there were more smokers than in the control group (*P*=0.006). Hypertension, coronary heart disease, and diabetes are the main clinical comorbidities. Hypertension is more common in patients with moderate to severe OSAHS (*P* < 0.001). As a major risk factor for OSAHS, the BMI of patients with moderate to severe OSAHS was significantly higher than that of patients with mild OSAHS and normal subjects (*P* < 0.001). The Epworth Sleepiness Scale score in the non-/mild OSAHS group was significantly lower than that in the moderate-to-severe OSAHS group (*P* < 0.001), suggesting that OSAHS patients with moderate or higher OSAHS have a clear tendency for subjective daytime sleepiness. According to the definition of AHI, the AHI value and oxygen reduction index (ODI) of the moderate-to-severe OSAHS group were significantly higher than those of the control group (*P* < 0.001); the average transcutaneous oxygen saturation (MSpO_2_) and the minimum transcutaneous oxygen saturation (LSpO_2_) were lower in patients with moderate to severe OSAHS (*P* < 0.001). The proportion of stage 1 sleep in patients with moderate to severe OSAHS (*P*=0.674) was comparable to that of the control group, and the proportion of stage 2 (*P*=0.005) light sleep was increased, while the proportion of stage 3 deep sleep (*P*=0.009) to REM (rapid eye movement) sleep (*P*=0.119) ratio is significantly reduced. Patients with moderate to severe OSAHS fell asleep faster than the control group; that is, the latency to fall asleep was significantly shorter (*P* < 0.001). The prevalence of different age groups is shown in Figure 6.

Increased CPAP assists in controlling blood pressure while treating OSAHS and significantly reduces the patient's 24 h average diastolic blood pressure and 24 h average arterial pressure (2.62 mmHg, *P*=0.019, and 2.70 mmHg, *P*=0.030); the 24-hour average arterial pressure was 2.62 mmHg, *P*=0.019 and 2.70 mmHg, *P*=0.030); although the 24-hour average systolic blood pressure improved slightly, but the difference was not statistically significant (2.8 mmHg, *P*=0.078). After 30 days of CPAP treatment, the patients' mean systolic blood pressure at night (5.61 mmHg, *P*=0.008) and morning peak mean systolic blood pressure (6.26 mmHg, *P*=0.010) were significantly reduced, and the difference was statistically significant. The PSG measurement results are shown in Table 3.

There were significant differences in AHI, LSpO_2_ (%), BMI, and other indicators in 14 cases before and after treatment with CPAP alone, *P* < 0.01. After treatment, the symptoms of snoring and holding breath were significantly reduced and blood oxygen saturation increased to varying degrees. The proportion of AHI, LSpO_2_ (%), and BMI indicators is shown in Figure 7.

## 5. Conclusion

The information storage function of the smart positive pressure ventilator is contained in the local medical terminal, presented after logging in with the user authority, and it is mainly composed of data collection, data processing, and medical interface design. When the CPAP ventilator transmits respiratory data to the local medical terminal, it sends real-time respiratory information data packets. The data packet is collected and sent in real time in a fixed period and then received and analyzed by the local medical terminal. In the CPAP ventilator telemedicine system, the function of alarm message processing is mainly to detect the patient's breathing status in real time, extract the alarm-related information, and generate an alarm. This study may help improve the quality of life of patients with obstructive sleep apnea syndrome. In the future work, the exhalation resistance can be reduced at the initial exhalation of the ventilator and the patient's comfort can be increased. A higher positive end-expiratory pressure can be given at the end of the expiration, which can prevent the patient from breathing at the end of each exhalation. The tract collapses to keep the airway open, which can greatly improve the patient's sleep quality, thereby ensuring the effectiveness of the treatment and the comfort of the patient. At present, the positive pressure mask cannot adjust the exhalation resistance, so it is possible to design a device that can adjust the initial pressure of the exhalation through the exhalation flow to achieve the therapeutic effect and improve the comfort of the patient.

## Figures and Tables

**Figure 1:** Positive pressure ventilator (http://alturl.com/afqj5).

**Figure 2:** The principle of operation of a smart positive pressure ventilator.

**Figure 3:** Logistic analysis results.

**Figure 4:** Measurement results of each index of the subject.

**Figure 5:** Pearson correlation analysis results.

**Figure 6:** The prevalence of different age groups.

**Figure 7:** The proportion of AHI, LSpO_2_ (%), and BMI indicators.

**Table 1:** Treatment status of each group.

Group	(Male/female) example	Age (years, *x* ± *S*)	BMI (kg/m^2^, *X* ± *S*)
Application group	22/11	50 ± 26	27.2 ± 5.5
Deprecated group	31/5	50 ± 21	29.1 ± 7.1
*P* value	0.056	0.101	0.595

**Table 2:** Changes of indicators before and after treatment.

Group	Before treatment	After treatment	*t*	*P*
BMI (kg/m^2^)	28.40 ± 3.74	27.75 ± 3.38	1.813	0.068
Neck circumference (cm)	39.61 ± 4.40	39.27 ± 4.18	1.041	0.300
Waist circumference (cm)	97.56 ± 9.63	97.26 ± 7.93	1.226	0.223
Hip circumference (cm)	103.84 ± 6.69	103.65 ± 6.79	1.453	0.149
FG (mmol/L)	5.71 ± 1.15	5.75 ± 1.11	−1.429	0.156
TC (mmol/L)	4.74 ± 0.93	4.43 ± 0.94	1.145	0.255

**Table 3:** PSG measurement results.

MAMS	PSG		Total
	+	−	
+	67 (95.7%)	3 (4.3%)	70
−	0 (0%)	2 (5.4%)	2
Total	67	5	73

## Data Availability

No data were used to support this study.
